This article has been retracted.

# Antitumor Activity of Sorafenib in Human Cancer Cell Lines with Acquired Resistance to EGFR and VEGFR Tyrosine Kinase Inhibitors

**DOI:** 10.1371/journal.pone.0028841

**Published:** 2011-12-09

**Authors:** Floriana Morgillo, Erika Martinelli, Teresa Troiani, Michele Orditura, Ferdinando De Vita, Fortunato Ciardiello

**Affiliations:** Division of Medical Oncology, Department of Clinical and Experimental Medicine and Surgery "F. Magrassi e A. Lanzara" Second University of Naples, Naples, Italy; Consiglio Nazionale delle Ricerche (CNR), Italy

## Abstract

Treatment of non small cell lung cancer (NSCLC) and colorectal cancer (CRC) have substantially changed in the last years with the introduction of epidermal growth factor receptor (EGFR) inhibitors in the clinical practice. The understanding of mechanisms which regulate cells sensitivity to these drugs is necessary for their optimal use.

An in vitro model of acquired resistance to two tyrosine kinase inhibitors (TKI) targeting the EGFR, erlotinib and gefitinib, and to a TKI targeting EGFR and VEGFR, vandetanib, was developed by continuously treating the human NSCLC cell line CALU-3 and the human CRC cell line HCT116 with escalating doses of each drug. MTT, western blot analysis, migration, invasion and anchorage-independent colony forming assays were conducted in vitro and experiments with established xenografts in athymic nude mice were performed in vivo in sensitive, wild type (WT) and TKI-resistant CALU-3 and HCT116 cell lines.

As compared to WT CALU-3 and HCT116 human cancer cells, TKI-resistant cell lines showed a significant increase in the levels of activated, phosphorylated AKT, MAPK, and of survivin. Considering the role of RAS and RAF as downstream signals of both the EGFR and VEGFR pathways, we treated resistant cells with sorafenib, an inhibitor of C-RAF, B-RAF, c-KIT, FLT-3, RET, VEGFR-2, VEGFR-3, and PDGFR-β. Sorafenib reduced the activation of MEK and MAPK and caused an inhibition of cell proliferation, invasion, migration, anchorage-independent growth in vitro and of tumor growth in vivo of all TKI-resistant CALU-3 and HCT116 cell lines.

These data suggest that resistance to EGFR inhibitors is predominantly driven by the RAS/RAF/MAPK pathway and can be overcame by treatment with sorafenib.

## Introduction

The epidermal growth factor receptor (EGFR) is a central regulator of cancer cell proliferation and progression in several human cancer types. The clinical efficacy of EGFR inhibitors (cetuximab, panitumumab, erlotinib, gefitinib and vandetanib) introduced in the clinical practice for the treatment of metastatic cancers is limited to a subgroup of patients with the majority of cancer patients showing either intrinsic or acquired resistance to these drugs [1].

The recent progresses in the knowledge of cancer biology and drug-resistance mechanisms have identified, among the intracellular signalling pathways, that act as down-stream to the EGFR, the AKT and RAS/RAF/ mitogen-activated protein kinase (MAPK) pathways as major responsible for the development of cancer cell resistance to EGFR inhibitors [2]–[4].

However, we recently demonstrated that, in our in vitro non small cell lung cancer (NSCLC) model of acquired resistance to erlotinib and gefitinib, treatment with several agents known to target directly or indirectly the AKT signalling pathway, such ad LY294002, deguelin and everolimus, was not efficacious in inhibiting erlotinib- (ERL-) and gefitinib- (GEF-) resistant cancer cell proliferation [5].

On the other side, mutations of the K-RAS gene has been described both in NSCLC and colorectal cancer (CRC) patients as responsible for a poor prognosis and poor response to EGFR inhibitors [6]. These mutations cause KRAS proteins to accumulate in the GTP-bound, active form leading to constitutive, growth-factor-receptor independent activation of KRAS downstream signaling in tumor cells [7]. The development of therapeutic strategies for patients with KRAS mutations is thus an important clinical goal. RAF serine-threonine kinases are the principal effectors of RAS in the MAPK signaling pathway and is therefore a potential target for cancer therapy. To date, the most successful clinical inhibitor of RAF activity is sorafenib (Nexavar, BAY 43-9006) [8]–[10], an orally available multi-targeted kinase inhibitor, that blocks the activation of C-RAF, B-RAF (both the wild-type and the activated V600E mutant), c-KIT, FLT-3, RET, vascular endothelial growth factor receptor 2 (VEGFR-2), VEGFR-3, and platelet-derived growth factor receptor β (PDGFR-β) [8]–[10], currently approved for the treatment of metastatic renal cell carcinoma (RCC) and for advanced hepatocellular carcinoma (HCC), and under investigation in other malignancies. Sorafenib affects tumor growth by directly inhibiting tumor cell proliferation and promoting apoptosis in a variety of tumor types as well as by inhibiting tumor-induced neoangiogenesis.

Our laboratory has recently provided evidence of a synergistic interaction between sorafenib and erlotinib or between sorafenib and cetuximab, a monoclonal antibody targeting the extracellular domain of the EGF receptor, in a panel of NSCLC and colorectal cancer (CRC) cell lines, *in vitro* and *in vivo*, which is accompanied by a marked and sustained inhibition of the MAPK- and AKT-dependent intracellular signals [11].

We hypothesized that treatment with sorafenib could overcome the induced EGFR TKI-resistance by its ability to block several growth factor receptor-driven signals. Moreover, because sorafenib blocks B-RAF, and it could be effective in cancer cell lines expressing activating K-RAS mutations.

In the present study, we report on the development and on the characterization of human NSCLC and CRC cell lines with acquired resistance to two tyrosine kinase inhibitors (TKI) targeting the EGFR, erlotinib and gefitinib, and a TKI targeting EGFR, VEGFR and RET, vandetanib, and on the antitumor effects of sorafenib in these resistant cancer cell lines.

## Results

### Development and characterization of TKI-resistant CALU-3 and HCT116 cancer cells

The human NSCLC CALU-3 cell line and the human CRC HCT116 cell line harbour the wild type EGFR gene and an activating K-RAS (KRASp.G13D) gene mutation. In contrast to the other K-RAS mutations, this mutation has been described as not influencing the sensitivity to anti-EGFR treatment, in particular cetuximab [11]. These cancer cell lines has been previously characterized by our group for the expression of the four EGF-related growth factor receptors (EGFR, ERBB2, ERBB3, and ERBB4) and of three VEGF receptors (VEGFR-1,VEGFR-2, VEGFR-3), as well as for the expression of three EGFR ligands (amphiregulin, EGF, and TGFα) and of three VEGFR ligands (VEGF-A, VEGF-B, VEGF-C), by using quantitative RT-PCR (qRT-PCR) [12]. All tested ligand mRNAs were expressed in CALU-3 and HCT116 cell lines. CALU-3 cells also expressed EGFR mRNA, whereas low levels of ERBB2 and ERBB3 mRNAs were measurable. VEGFR-2 and VEGFR-3 mRNA expression was detected in CALU-3 cell line. Expression of EGFR and its specific ligands suggests that in these human cancer cell lines an EGFR-driven autocrine pathway is relevant for cancer cell proliferation. In fact, CALU-3 and HCT116 cells are growth-inhibited by treatment with selective EGFR TKIs, such as gefitinib or erlotinib [13]. Furthermore, these cancer cells express both VEGF ligands and VEGFRs and are growth inhibited by treatment with anti-angiogenic TKIs [13].

Therefore, CALU-3 and HCT116 cells were selected as a model for exploring the acquired resistance mechanisms to treatment with the EGFR TKIs erlotinib and gefitinib, or with the dual EGFR/VEGFR tyrosine kinase inhibitor vandetanib.

The gefitinib- (GEF-R), erlotinib- (ERL-R) and vadetanib- (VAN-R) resistant cell lines were obtained by continuously culturing CALU-3 and HCT116 cells in the presence of increasing doses of each drug for 12 months. After the establishment of three different TKI-resistant CALU-3 and three different TKI-resistant CALU-3 HCT116 cell lines, we characterized their resistant phenotype by doing cell proliferation assays in the presence of each of these inhibitors. As illustrated in Table 1, an approximately 10-fold increase in the IC_50_ for each TKI-resistant cell line as compared with parental cells was observed. ERL-R, GEF-R and VAN-R CALU-3 and HCT116 human cancer cell lines were cross-resistant to either gefitinib, erlotinib or vandetanib treatment. We next confirmed the establishment of stable TKI-resistant CALU-3 and HCT116 cancer cells in a drug-free culture medium. In fact, all six TKI-resistant cell lines could grow in the absence of each drug for long periods of time (three to six months) and maintain their TKI-resistant phenotype (data not shown).

**Table 1:** IC50 for treatment with erlotinib, gefitinib or vandetanib in parental CALU-3 and HCT116 cell lines (WT) and their TKI-resistant derivatives (ERL-R, GEF-R, VAN-R).

	CALU-3				HCT116			
	WT	ERL-R	GEF-R	VAN-R	WT	ERL-R	GEF-R	VAN-R
ERLOTINIB	3 µM	≥25 µM	≥25 µM	≥25 µM	7 µM	≥25 µM	≥25 µM	≥25 µM
GEFITINIB	6 µM	≥25 µM	≥25 µM	≥25 µM	10 µM	≥25 µM	≥25 µM	≥25 µM
VANDETANIB	5 µM	≥25 µM	≥25 µM	≥25 µM	6 µM	≥25 µM	≥25 µM	≥25 µM

To further characterize the TKI-resistant CALU-3 and HCT116 cell lines, we examined differential protein expression among wild type, sensitive CALU-3 and HCT116 cells and their TKI-resistant derivatives.

Activation of the EGFR leads to a complex intracellular signalling which includes the activation of the pro-survival PI3K/AKT pathway and the mitogenic RAS/RAF/MEK/MAPK pathway [13], [14]. We, therefore, investigated by immunoblotting analysis these molecular pathways. As illustrated in Figure 1, EGF-stimulated activation of the EGFR was efficiently blocked in WT and ERL-R, GEF-R and VAN-R cells as demonstrated by the inhibition of EGFR auto-phosporylation (P-EGFR).

**Figure 1:** Analysis of EGFR downstream pathways in parental CALU-3 and HCT116 cells (WT) and in their TKI-resistant derivatives 8ERL-R, GEF-R, VAN-R). Western blotting analysis of EGFR and of down-stream signalling pathways in parental human CALU-3 and HCT116 cells (WT) and in their TKI-resistant derivatives (ERL-R, GEF-R, VAN-R). β-actin was included as a loading control.

Since the activated, phosphorylated forms of AKT and MAPK are key intracellular mediators of growth factor-activated cell survival and proliferation signals [13], [14] investigating the activation state of these molecular pathways may be of interest in the understanding the resistance mechanisms. Activation of MAPK and AKT with an increase in their phosphorylated forms (P-MAPK and P-AKT) as well as an increase in survivin protein levels were observed in all three TKI-resistant CALU-3 cell lines and in all three TKI-resistant HCT116 cell lines as compared to their parental counterpart (Figure 1).

Taken together, these results suggest that in this cancer cell model of acquired resistance to three different TKIs, activation of AKT- and MAPK-driven intracellular signals may be responsible for cancer cell growth in the presence of either selective anti-EGFR TKIs, such as gefitinib or erlotinib, or in the presence of broad spectrum TKI, such as vandetanib.

### Effects of sorafenib on TKI-resistant CALU-3 and HCT116 cancer cell growth

In light of the role of RAS and RAF as downstream mediators of both the EGFR and VEGFR signals from cell surface, we tested the anti-proliferative effect of sorafenib, a multi-targeted kinase inhibitor, blocking the activation of C-RAF, B-RAF, c-KIT, FLT-3, RET, VEGFR-2, VEGFR-3, and PDGFR-β [8] on the parental WT and TKI-resistant CALU-3 and HCT116 cancer cells. A significant inhibition of cell growth was observed in both WT CALU-3 cells and WT HCT116 cells and their corresponding three TKI-resistant derivatives following sorafenib treatment, with an IC_50_ ranging from 0. 1 to 0.5 µM, (Figure 2).We further characterized the effects of sorafenib treatment on intracellular signalling by Western blotting. As illustrated in Figure 3, treatment of ERL-R, GEF-R and VAN-R CALU-3 and HCT116 cells with sorafenib for 48 hours did not affect total MEK and MAPK protein levels, while it caused a marked decrease of the phosphorylated, activated forms of MEK (P-MEK) and of MAPK (P-MAPK). Moreover, we investigated the activation status of all molecular targets of sorafenib by studing the protein expression levels of C-RAF, B-RAF, c-Kit, FLT-3, RET, VEGFR-2, VEGFR-3 and PDGFRβ, and their phosphoryation status by western blotting analysis. Among all the targets of sorafenib activity, only C-RAF and B-RAF resulted activated in resistant CALU-3 and HCT116 cancer cell lines, and therefore strongly inhibited by sorafenib treatment (Figure 3).

**Figure 2:** Growth inhibitory effects of treatment with sorafenib in parental and TKI-resistant CALU-3 and HCT116 cancer cells. MTT cell proliferation assays were performed in parental lung adenocarcinoma CALU-3 and colorectal cancer HCT116 cells. (WT) and in their TKI-resistant derivatives (ERL-R, GEF-R, VAN-R ), treated for three days with the indicated concentrations of sorafenib. Results represent the average (±SD) of three separate experiments, each performed in quadruplicate.

**Figure 3:** Western blotting analysis of CALU-3 and HCT116 cells TKI-resistant derivatives (ERL-R, GEF-R, VAN-R) following treatment with sorafenib. Western blotting analysis of C-RAF, B-RAF, MEK and MAPK activation following treatment with the indicated concentration of sorafenib of lung adenocarcinoma CALU-3 and colorectal cancer HCT116 cells TKI-resistant derivatives (ERL-R, GEF-R, VAN-R ). β-actin was included as a loading control.

### Effects of sorafenib treatment on the invasion, migration and anchorage-independent growth of TKI-resistant CALU-3 and HCT116 cancer cells

It has been suggested that cancer cells undergoing resistant to anti-EGFR drugs could gain a more aggressive and metastatic phenotype with increased ability to invade, migrate and to form colonies in semisolid medium [15]. Therefore, we evaluated these properties in TKI-sensitive WT CALU-3 and HCT116 cancer cells and in their TKI-resistant derivatives. As illustrated in Figure 4, WT CALU-3 and HCT116 cells demonstrated little or no ability in invasion and migration. On the contrary, all TKI-resistant CALU-3 and HCT116 cell lines exhibited significant invasive and migratory abilities. Moreover, their anchorage-independent colony growth was increased of approximately 3-fold as compared to WT cells (Figure 4). Collectively, these results suggest that cancer cell lines with acquired resistance to erlotinib, gefitinib and vandetanib have acquired a more invasive and, potentially, more metastatic behaviour.

**Figure 4:** Effects of treatment with sorafenib on the invasive, migratory and anchorage-independent colony forming capabilities of TKI-resistant CALU-3 and HCT116 cancer cells. Anchorage-independent growth (A), migration (B) and invasion (C), were evaluated in TKI-resistant CALU-3 and HCT116 derivatives (ERL-R, GEF-R, VAN-R) after treatment with the indicated concentrations of sorafenib. The results are the average ± SD of three independent experiments, each done in triplicate. Representative pictures are shown for the migration and invasion abilities of CALU-3 WT and Resistant cell lines.

We next evaluated the effects of sorafenib on the invasive and migratory capabilities of the TKI-resistant CALU-3 and HCT116 cell lines. We did not tested the effect of sorafenib treatment on TKI-sensitive WT cancer cell lines in consideration of the absence of migratory and invasive ability. A significant dose-dependent inhibition of invasion and migration was observed in all TKI-resistant cell lines following treatment with sorafenib (Figure 4).

### Effects of sorafenib on TKI-resistant CALU-3 and HCT116 tumor xenografts

We finally investigated the in vivo antitumor activity of sorafenib in nude mice bearing WT CALU-3 and HCT116 or TKI-resistant CALU-3 and HCT116 cell lines which were grown subcutaneously as xenografts. In WT CALU-3 and HCT116 tumor xenografts, treatment with sorafenib caused a significant decrease in tumor size as compared to control untreated mice. For example, at day 35 from the starting of treatment, the mean tumor volume in mice bearing WT tumor xenografts and treated with sorafenib was respectively 38% and 31% in CALU-3 and HCT116 as compared to control untreated mice (Figure 5, 6). Also in mice bearing ERL-R, GEF-R or VAN-R CALU-3 and HCT116 tumor xenografts, treatment with sorafenib induced a significant reduction in tumor growth (Figure 5, 6). In this respect, at day 35 from the starting of treatment, the mean tumor volumes in the sorafenib-treated mice ranged between 27% and 40%, as compared to control untreated mice.

**Figure 5:** Antitumor activity of the sorafenib in parental and TKI-resistant CALU-3 xenografts. A, Parental (WT) CALU-3 cancer cells; B, GEF-R CALU-3 cancer cells; C, VAN-R CALU-3cancer cells; D, ERL-R CALU-3 cancer cells. Athymic nude mice were injected subcutaneously into the dorsal flank with 10^7^ cancer cells. After 7 to 10 days (average tumor size, 75 mm^3^), mice were treated as indicated in Materials and Methods for 5 weeks. Each treatment group consisted of 8 mice. Data represent the average (±SD). Student's *t* test was used to compare tumor sizes among different treatment groups at day 35 following the start of treatment. A, CALU-3 WT: sorafenib versus control (two-sided p<0.001); B, CALU-3 GEF-R: sorafenib versus control (two-sided p<0.001). C, CALU-3 VAN-R: sorafenib versus control (two-sided p<0.001); D, CALU-3 ERL-R: sorafenib versus control (two-sided p<0.001).

**Figure 6:** Antitumor activity of the sorafenib in parental and TKI-resistant HCT116 xenografts. A, Parental (WT) HCT116 cancer cells; B, GEF-R HCT116 cancer cells; C, VAN-R HCT116 cancer cells; D, HCT116 cancer cells. Athymic nude mice were injected subcutaneously into the dorsal flank with 10^7^ cancer cells. After 7 to 10 days (average tumor size, 75 mm^3^), mice were treated as indicated in Materials and Methods for 5 weeks. Each treatment group consisted of 8 mice. Data represent the average (±SD). Student's *t* test was used to compare tumor sizes among different treatment groups at day 35 following the start of treatment. A, HCT116 WT: sorafenib versus control (two-sided p<0.001); B, HCT116: sorafenib versus control (two-sided p<0.001). C, HCT116 VAN-R: sorafenib versus control (two-sided p<0.001); D, HCT116 ERL-R: sorafenib versus control (two-sided p<0.001).

## Discussion

Activation of the EGFR and the VEGFR pathways play a key role in the development and progression of the majority of epithelial cancers including NSCLC and CRC. However, only a subgroup of patients benefits of treatments with drugs targeting the EGFR or the VEGFR pathways [16]. Indeed, even in initially responding patients secondary or acquired resistance occurs causing cancer progression and treatment failure. Several molecular mechanisms have been suggested to explain the acquisition of cancer cell resistance to molecularly targeted anti-cancer drugs [16].

Cancer cell resistance to EGFR antagonists could be due to several reasons. Host related mechanisms, such as defective immune-system activity, rapid metabolism or poor absorption, are responsible for intrinsic or primary resistance. Moreover, the genetic instability of these cells generates cancer cell clones with an acquired resistance following prolonged exposure to EGFR inhibitors. Since EGFR antagonists interfere with the activation of several intracellular pathways that control cell proliferation, survival, apoptosis, metastatic capability, invasion and tumor-induced angiogenesis, it is clear that several different molecular changes could be responsible for the development of resistance to these inhibitors [16].

In the present study, we found that cancer cells which develop resistance to the EGFR tyrosine kinase inhibitors following long time treatment (acquired resistance) exhibit activated RAS/RAF/MAPK and AKT pathways. The EGFR-independent activation of these downstream pathways makes cancer cells insensitive to the EGFR inhibition and represents one of the most common reported causes of resistance to EGFR-targeted therapy in solid tumors.

The constitutive activity of at least one of these two pathways has been demonstrated to be able to defines a resistant phenotype unaffected by the treatment with gefitinib and cetuximab [2], [17].

Persistent phosphorylation of the RAS/RAF/MAPK and/or AKT pathways can be explained with the activation of cell surface receptors other than EGFR such as insulin-like growth factor-1 receptor (IGF-1R) and MET [18]–[21], which are known to be iperexpressed or activated in the presence of persistent inhibition of the EGFR.

Moreover, an increased receptor-independent activity of the RAS/RAF/MAPK and/or AKT pathways could results from direct gene amplification, activating/inactivating mutations or loss of molecular regulator [22], [23].

However, whereas inhibition of the AKT pathway does not interfere with the proliferation of resistant cells, the inhibition of the RAF/MEK/MAPK pathway by sorafenib treatment strongly reduces cell growth and survival. Indeed, among all the molecular targets of sorafenib, only C-RAF and B-RAF resulted activated in resistant cell lines probably by upstream receptors not yet tested in this work; however this information suggests that the activation of RAF-dependent intracellular signals could be an important mechanism in the acquisition of resistance to anti-EGFR therapy.

The RAS/RAF/MAPK signaling pathway is a promising therapeutic target given its central role in regulation of mammalian cell proliferation, relaying extracellular signals from ligand-bound receptor tyrosine kinases at the cell surface to the nucleus via a cascade of specific phosphorylation events. The mutational status of RAS and B-RAF genes has been demonstrated to affect the sensitivity of tumor cell lines to inhibitors of the EGFR [24]. However, therapeutic targeting of the RAS pathway has so far been unsuccessful. RAF serine-threonine kinases are the principal effectors of RAS and are considered an important target for cancer therapy. Agents such as sorafenib that bypass RAS and inhibit effector molecules downstream of the mutant GTPase (e.g. RAF) are being evaluated. Preclinical data have suggested that sorafenib inhibits cell growth by inducing G1 arrest in NSCLC cell lines independent of KRAS genotype [8].

Another possible mechanism of resistance to the EGFR inhibition may be an increased angiogenic potential through enhanced endothelial cell proliferation and permeabilization. On the basis of this informations, several preclinical studies have been realized with the intent to discover the effects of a combined targeting of the erbB and VEGF pathways by using different approaches [25]–[29]. In addition to the option of using anti- EGFR therapies in combination with anti-VEGF drugs, a series of tyrosine kinases that block both the EGFR and the VEGF receptor TK were developed, such as vandetanib, which has demonstrated significant activity as single agent and in combination with traditional chemotherapeutics in several human tumor types [27]–[29].

Often, EGFR inhibitor-resistant human cancer cell lines exhibit, as common feature, VEGFR overexpression, increased secretion of VEGF and placental growth factor, and augmented migration capabilities. Sorafenib inhibits several RTKs that participate in neovascularization, including vascular endothelial growth factor receptor (VEGFR)-2 and VEGFR-3 [30]. Inhibition of angiogenesis might thus be expected to contribute to the inhibition of tumor growth by this drug in addition to its effects on RAF signaling. Although sorafenib was previously shown to inhibit the growth of a variety of human tumor xenografts in mice [8], it has been difficult to measure the relative contributions of its antiangiogenic activity and its direct antitumor activity mediated by RAF inhibition. Moreover, in our work, the development of human cancer cells resistant to vandetanib, excluded the possibility that sorafenib'efficacy may depend on the inhibition of the VEGFR.

Evidence of a positive interaction between sorafenib and anti-EGFR drugs have recently been provided by our group [12]. Preclinical evidences supported a strong anti-proliferative and anti-migratory effects in NSCLC and CRC cancer cell lines following the combination with sorafenib plus ant-EGFR drugs [12]. Moreover, a recent phase II clinical study supported the combination of erlotinib and sorafenib in elderly patients with advanced NSCLC in light of the higher 1-year survival rate [30].

In the present study, we have provided evidences that sorafenib is active in inhibiting tumor cell growth *in vitro* and *in vivo* of human cancer cells resistant to inhibitor of the EGFR and/or VEGFR. The activity of sorafenib is strictly linked to its ability to block RAF signaling through the RAS/RAF/MEK/MAPK pathway.

## Methods

### Cell lines, drugs and chemicals

The human NSCLC CALU-3 and the human CRC HCT116 cell lines were provided by the American Type Culture Collection (Manassas, VA) and maintained in RPMI 1640 supplemented with 10% fetal bovine serum (FBS; Life Technologies, Gaithersburg, MD) in a humidified atmosphere with 5% CO_2_. Gefitinib and vandetanib were provided by AstraZeneca, Macclesfield, UK; erlotinib was provided by Roche, Basel, Switzerland; sorafenib was provided by Bayer Schering Pharma, Leverkusen, Germany. Primary antibodies against P-EGFR (Tyr1173), EGFR, P-MAPK44/42 (Thr202/Tyr204), MAPK44/42, P-AKT (Ser473), AKT, P-MEK (Ser217/221), MEK, P-B-RAF (ser 445), P- C-RAF (ser 338), survivin were obtained from Cell Signaling Technology, Danvers, MA, USA. Cell invasion and migration assay kits were obtained by Chemicon, Millipore, CA, USA. All other chemicals were purchased from Sigma Aldrich, MO, USA.

### Establishment of CALU-3 and HCT116 cancer cell lines with acquired resistance to different TKIs

Over a period of 12 months, human CALU-3 lung adenocarcinoma cells and human HCT116 colorectal carcinoma cells were continuously exposed to increasing concentrations of either gefitinib, erlotinib or vandetanib, as previously described (12). The starting dose was the dose causing the inhibition of 50% of cancer cell growth (IC_50_) for each EGFR inhibitor (i.e.: erlotinib, 3 µM; gefitinib, 6 µM; vandetanib, 1 µM). The drug dose was progressively increased to 15 µM in approximately two months, to 20 µM after other two months, to 25 µM after additional two months, and, finally, to 30 µM for a total of 12 months. The established resistant cancer cell lines were then maintained in continuous culture with the maximally achieved dose of each TKI that allowed cellular proliferation (30 µM for each drug).

### Cell proliferation assay

Cancer cells were seeded in 96-well plates and were treated with different drugs, such as erlotinib, gefitinib, vandetanib or sorafenib for 72 hours. Cell proliferation was measured with the 3-(4,5-dimethylthiazol-2-yl)-2,5-diphenyltetrazolium bromide (MTT) assay. The IC_50_ were determined by interpolation from the dose-response curves. Results represents the median of three separate experiments each performed in quadruplicate.

### Western blotting analysis

Following treatment, cancer cells were lysed with Tween-20 lysis buffer (50 mmol/L HEPES, pH 7.4, 150 mmol/L NaCl, 0.1% Tween-20, 10% glycerol, 2.5 mmol/L EGTA, 1 mmol/L EDTA, 1 mmol/L DTT, 1 mmol/L phenylmethylsulfonylfluoride, and 10 µg/mL of leupeptin and aprotinin) and sonicated. Equal amounts of protein were analyzed by SDS-PAGE. Thereafter, proteins were transferred to nitrocellulose membranes and analyzed by specific primary antibodies, as indicated in the experiment. Proteins were detected via incubation with horseradish peroxidase–conjugated secondary antibodies and ECL chemiluminescence detection system.

### Invasion assay

The invasive ability in vitro was measured by using transwell chambers, according to the manufacturer's protocol. Briefly, cells were seeded onto the membrane of the upper chamber of the transwell at a concentration of 2×10^5^/ml in 500 µl of RPMI medium and were left untreated or treated with the indicated doses of sorafenib for 24 hours. The medium in the upper chamber was serum-free. The medium at the lower chamber contained 10% FBS as a source of chemo-attractants. Cells that passed through the Matrigel coated membrane were stained with Cell Stain Solution containing crystal violet supplied in the transwell invasion assay (Chemicon, Millipore, CA) and photographed after 20 hours of incubation. Absorbance was measured at 562 nm by an ELISA reader after dissolving of stained cells in 10% acetic acid. Assays were performed in triplicate.

### Migration assay

Cell migration was assessed using a commercially available chemotaxis assay. Briefly, cells were incubated in RPMI serum-free medium for 24 hand were left untreated or treated with the indicated doses of sorafenib, following which they were detached from flasks, suspended in quenching medium (serum-free medium containing 5% bovine serum albumin) and EDTA, and seeded into Boyden migration chamber inserts placed in a 24-well plate. The inserts contain a microporous membrane with an 8-µm pore size. Inserts were placed over wells containing serum-free media plus chemo-attractant (10% FBS). After a 48-h treatment period, cells/media were discarded from the top side of the migration chamber insert and the chamber was placed in the wells of a new 24-well plate containing cell detachment solution. Following incubation for 30 min at 37°C, the insert was discarded, and a solution of lysis buffer and CyQuant GR dye was added to each well. CyQuant is a green fluorescent dye that exhibits strong enhancement of fluorescence when bound to cellular nucleic acids released by the lysis buffer, enabling assessment of the relative number of migrated cells. Fluorescence was determined with a fluorimeter at 480/520 nm. Assays were performed in triplicate.

### Growth in soft agar

Cells (10^4^ cells/well) were suspended in 0.5 mL 0.3% Difco Noble agar (Difco, Detroit, MI) supplemented with complete culture medium. This suspension was layered over 0.5 mL 0.8% agar-medium base layer in 24 multiwell cluster dishes (Becton Dickinson, Lincoln Park, NJ) and treated with different concentrations of sorafenib. After 14 days, cells were stained with nitro blue tetrazolium (Sigma, St. Louis, MO) and colonies larger than 0.05 mm were counted. Assays were performed in triplicate.

### Tumor xenografts in nude mice

Four- to six-week old female balb/c athymic (nu+/nu+) mice were purchased from Charles River Laboratories (Milan, Italy). The research protocol was approved by the Second University of Naples Animal Care and Use Committee (IT2010/20299). Mice were maintained in accordance with the institutional guidelines of the Second University of Naples Animal Care and Use Committee. Mice were acclimatized for one week prior to being injected with cancer cells and injected subcutaneously with 10^7^ CALU-3 (WT, ERL-R, GEF-R, or VAN-R) cells or with 10^7^ HCT116 (WT, ERL-R, GEF-R, or VAN-R) cells, that had been resuspended in 200 µL of Matrigel (Becton Dickinson). When established tumors of approximately 75 mm^3^ in diameter were detected, mice were treated with oral administrations of sorafenib (50 mg/kg/day), for the indicated time periods. Each treatment group consisted of 8 mice. Tumor volume was measured using the formula π/6 x larger diameter x (smaller diameter)^2^.

### Statistical analysis

The Student's t test was used to evaluate the statistical significance of the results. All P values represent two-sided tests of statistical significance. All analyses were performed with the BMDP New System statistical package version 1.0for Microsoft Windows (BMDP Statistical Software, Los Angeles, CA).
